# A Systematic Review and Meta-Analysis of the Relationship between Receiving the Flu Vaccine with Acute Cerebrovascular Accident and Its Hospitalization in the Elderly

**DOI:** 10.1155/2023/2606854

**Published:** 2023-02-13

**Authors:** Nilay Rezaei Tavabe, Soleiman Kheiri, Mohsen Dehghani, Abdollah Mohammadian-Hafshejani

**Affiliations:** ^1^Department of Epidemiology and Biostatistics, School of Health, Shahrekord University of Medical Sciences, Shahrekord, Iran; ^2^Department of Epidemiology, School of Public Health, Iran University of Medical Sciences, Tehran, Iran; ^3^Modeling in Health Research Center, Shahrekord University of Medical Sciences, Shahrekord, Iran

## Abstract

**Background and Aims:**

In recent years, various studies have been conducted worldwide to investigate the relationship between receiving the flu vaccine with acute cerebrovascular accident or stroke and its hospitalization in the elderly; however, the results of these studies are contradictory. Therefore, this study was aimed at investigating the relationship between receiving the flu vaccine with stroke and its hospitalization in the elderly.

**Methods:**

This study is a systematic review and meta-analysis of studies examining the relationship between receiving the flu vaccine with stroke and its hospitalization in the elderly during the years 1980 to 2021 which have been published in ISI Web of Science, Scopus PubMed, Cochrane, Science Direct, Google Scholar, and Embase. All analyses were performed by Stata 15, and the significance level in this study was considered <0.05.

**Results:**

In the systematic search, 3088 articles were retrieved, considering the study criteria; finally, 14 studies were included in the meta-analysis. Based on the results of the meta-analysis, the odds ratio (OR) of occurrence and hospitalization of stroke compared to the nonvaccinated group in vaccine recipients is equal to 0.84 (95% confidence interval (CI): 0.78-0.90, *P* value ≤ 0.001). Publication bias was not observed in this study (*P* value = 0.101).

**Conclusion:**

Getting the flu vaccine can reduce the risk of occurrence and hospitalization of stroke in the elderly by 16% (10%-22%). Therefore, receiving this vaccine as a preventive intervention for stroke in the elderly may be promising.

## 1. Introduction

Globally, the phenomenon of increasing life expectancy and the growing proportion of elderly people in the general population have led to the prevalence of chronic diseases [1–3]. Currently, the most important causes of death in most countries of the world include non-communicable diseases such as cardiovascular diseases, cancers, unintentional injuries, and strokes [4–8]. Acute cerebrovascular accident or stroke occurs when a factor blocks blood flow to a part of the brain or a blood vessel in the brain ruptures [9]. In this case, parts of the brain are damaged or die. Therefore, depending on the severity of the injury, stroke can cause permanent brain damage, long-term disability, or even death [10].

Stroke is one of the leading causes of morbidity and mortality in the world [11]; according to the World Health Organization (WHO), stroke is the second leading cause of death after heart disease, with more than seven million deaths in 2012, accounting for 11.1% of all deaths worldwide [12, 13]. In Europe, more than one million new strokes occur each year [14]. In the US, stroke is also considered to be one of the leading causes of death; however, the risk of stroke varies by race and ethnicity [15]. Blacks are almost twice as likely to have a stroke as whites, and blacks have the highest mortality rate. Although overall stroke mortality rates in the US are declining, Hispanics have seen an increase in deaths from the disease since 2013 [15]. The cost of stroke in the US from 2014 to 2015 was approximately $46 billion, including health care, stroke medications, and absenteeism. The American Heart and Stroke Association predicts that by 2030, direct medical costs for stroke will triple to $184.1 billion [16].

Stroke can occur at any age, and the risk of stroke increases with age [17]. In the US in 2009, 66% of patients admitted for stroke were over 65 years old [18]. Stroke is one of the leading causes of death in men [15], and men under the age of 44 are hospitalized with higher rates of ischemic stroke than women in the same age group [19].

To prevent stroke, it is important to identify and correct risk factors for the disease. In addition to the usual risk factors for stroke (i.e., aging, high blood pressure, smoking, diabetes, and high cholesterol), there is evidence that other risk factors, such as viral and bacterial infections, also play a role [20]. The incidence of cardiovascular disease (CVD), including stroke in winter and during influenza pandemics, is higher than at other times of the year [21], and changes in metabolic risk factors or vascular stress due to cold may be associated with the incidence of these diseases [22, 23]. However, there is ample evidence that influenza can be considered a trigger for CVD [24, 25]. A meta-analysis study by Barnes et al. [26] found that influenza infection was significantly associated with acute myocardial infarction (AMI) and similarly associated with stroke. Therefore, it is possible that immunization against influenza reduces the risk of CVD. The use of influenza vaccines in animal models to prevent CVD and AMI has had protective effects against the disease by reducing the size of atherosclerotic plaque, increasing plaque stability, and decreasing proinflammatory markers [27]. There is growing evidence that the flu vaccine is effective in preventing CVD [26, 28]. However, the association of influenza vaccines with stroke risk has been investigated in epidemiological studies, but their results are inconsistent. Some studies have shown that influenza vaccination is associated with a reduced risk of stroke [24, 29–31]. Conversely, the protective effects of the flu vaccine against CVD and acute cerebrovascular accidents have not been proven in some studies [32–34]. Therefore, there is no clear answer as to the relationship between the flu vaccine and the risk of stroke. Since one of the best ways to draw a definite conclusion and answer a scientific question is to use systematic review and meta-analysis studies, the present study uses the results of research studies conducted in this field with the method of a systematic review and meta-analysis to examine the association between receiving the flu vaccine and the risk of acute cerebrovascular accident or stroke and its hospitalization in the elderly. It can be stated that this systematic review and meta-analysis study is the most comprehensive and complete analysis of the relationship between receiving the flu vaccine with acute cerebrovascular accident and its hospitalization to date [35, 36], because it has been considered more recent and updated studies, and therefore, more participants and also subgroup analysis. In addition, this study is the only study that specifically evaluates the relationship between receiving influenza vaccine and the occurrence of stroke and its hospitalization in the elderly. Therefore, this study has provided a more convincing conclusion.

## 2. Materials and Methods

### 2.1. Type of Study and Population Studied

This study is a systematic review and meta-analysis conducted on the randomized clinical trials (RCTs), cross-sectional, case-control, or cohort studies that examine the association between receiving influenza vaccine and the occurrence of stroke and its hospitalization in the elderly between 1980 and July 2021.

### 2.2. Search Strategies

In this study, a comprehensive and complete search of studies published in ISI Web of Science, Scopus, PubMed, Cochrane, Science Direct, Google Scholar, and Embase databases was performed in the period from 1980 to July 2021. In this search, the criteria considered “influenza vaccine” as exposure and “occurrence of stroke” and “hospitalization” were considered as outcomes. Stroke is an acute illness, so hospitalization for a stroke can indicate new events. Therefore, in this study, hospitalization is considered an estimate of the occurrence of stroke.

To ensure access to all published studies in this regard, the reference list of articles retrieved in the electronic search was reviewed to access related studies. In the next step, by reviewing the titles, articles unrelated to the purpose of the research were excluded, and then among the remaining studies, by referring to the abstract and also the full text of the article, it was confirmed that it was relevant to the purpose of the study. Diagram 1 shows the process of identifying and selecting studies as well as how to examine them to enter into a systematic review and meta-analysis schematically.

### 2.3. Criteria for Inclusion and Exclusion of Studies

In this study, only studies performed by design such as RCTs, case-control, cross-sectional, and cohort studies were considered. Also, the effect size of the association between the influenza vaccine and the occurrence of stroke or hospitalization in the elderly should be considered in the article, or it should be calculated table based on the information in the article. Articles that did not provide sufficient data to calculate the effect size were excluded from the study. In addition, in this study, the searches were limited to studies that have been performed on humans. Also, only English language studies were considered.

### 2.4. Information Extracted from Studies

From the final articles included in this study, information such as study title, type of study, name of the first author, year of publication, country of study, the male-to-female of study participants, the age range of study participants, the average age of participants, sample size, number of people in vaccinated and nonvaccinated groups, duration of follow-up of participants, and relative risk, risk ratio, or odds ratio of a relationship between influenza vaccine and stroke or hospitalization with 95% CI as well as adjusted variables in a multivariate model, were extracted and collected.

### 2.5. Evaluation of the Quality of the Articles

Newcastle-Ottawa checklists were used to evaluate the quality of observational articles and Jadad for RCTs. Based on these checklists, the articles were divided into two categories: medium quality, and high quality. The quality of the articles was evaluated independently by two researchers and any differences were discussed with the third researcher.

### 2.6. Statistical Analysis

Due to the low incidence of the outcome under study (stroke occurrence or hospitalization due to stroke), the odds ratio estimated in various studies was considered an estimate of relative risk. In studies where the effect size was calculated and presented separately for time or seasonal periods, using the meta-analysis method, a total effect size was calculated from the presented values and considered in the analysis. Also, in studies where the effect size was not reported, but the information related to exposure and outcome was available, the effect size and its 95% CI were estimated.

The presence of heterogeneity in the studies included in the meta-analysis was assessed using statistical tests (chi-square test and *I*^2^ (to report a quantitative amount of heterogeneity)) and graphical methods (forest plot and Galbraith plot). Using the chi-square test, the heterogeneity in the results of the studies entered in the meta-analysis was investigated and the results of this test determined the type of model (fixed or random). To determine the factors related to heterogeneity in the results, the met-regression model was used by considering variables such as study sample size, article quality evaluation score, study design, follow-up period, year, age average of participants, sex ratio (male to female) of participants, and study location. Sensitivity analysis was also used to evaluate the effect of omitting each of the studies on the final result. Funnel diagrams and Begg's and Egger's tests were used for assessing publication bias. All analyses were performed by Stata statistical software (version 15.0, Stata Corp, College Station, TX), and the significance level in this study was considered <0.05.

## 3. Results

According to Figure 1, as of July 31, 2021, 3088 articles were retrieved in databases by keywords created in Mesh with title/abstract by electronic search, with repetition, 1592 articles were deleted, and 1496 articles remained in the study. By reviewing each article title, 939 articles in the title and abstract review and 515 articles in the full-text review were deleted. In the end, out of the remaining 42 articles, 13 articles were selected according to the criteria considered for the study. Finally, by reading the full text of these articles, one related article was extracted from the references mentioned in these articles and 14 articles were considered in the current systematic review and meta-analysis [24, 29–31, 37–46].

### 3.1. Characteristics of Selected Studies

In total, 14 studies were retrieved to investigate the relationship between receiving the flu vaccine and the risk of stroke or hospitalization. These studies were performed on 3,198,646 participants from 1995 to 2021 [24, 29–31, 37–46]. In terms of the geographical distribution of studies, 4 studies were conducted in Asia with a statistical population of 2,799,386 people (87.63%) [38, 41, 43, 46], 7 studies were conducted in Europe with a statistical population of 222,488 people (6.95%) [24, 29, 31, 39, 40, 44, 45], 2 studies were conducted in North America with a statistical population of 150,815 people (4.71%) [30, 37], and one study was conducted internationally with a statistical population of 22,837 people (0.71%) [42]. Eight of the studies were case-control studies [24, 29, 31, 37, 39, 40, 43, 44], and six studies were performed as cohorts [30, 38, 41, 42, 45, 46]. The range follow-up period of the participants is 6-84 months, and the average follow-up period is about 30 months (Tables 1 and 2).

### 3.2. Relationship between Receiving the Flu Vaccine with Stroke and Its Hospitalization

A review of 14 studies to determine the association between receiving the flu vaccine and the risk of stroke or hospitalization of the elderly due to stroke showed that compared to the elderly who did not receive the vaccine, the OR of having a stroke or being hospitalized in vaccine recipients is equal to 0.84 (95% CI:0.77-0.90, *P* value < 0.001). In other words, the results of this meta-analysis show that compared to the elderly who did not receive the flu vaccine, the odds of having a stroke or hospitalization in people receiving the flu vaccine decreased by 16% (10%-22%), which is also statistically significant (Figure 2).

### 3.3. Meta-regression and Sensitivity Analysis

To investigate the cause of heterogeneity in the results of studies, a meta-regression was performed in which the following variables were included: year, follow-up time, study type/design, sample size, quality of study based on the Newcastle-Ottawa, study period, age average of participants, sex ratio (male to female) of participants, and study location. The results from the meta-regression analysis determined there was no significant source of heterogeneity (*P* > 0.10). Moreover, sensitivity analysis was performed by excluding each study from the analysis one by one during each run. However, the estimated OR did not change significantly, further indicating the robustness of the meta-analysis results. (Table 3 and Figures 3 and 4).

### 3.4. Subgroup Analysis

To determine the reason for the heterogeneity, subgroup analysis was performed and studies based on sample size (more or less than 10,000 participants), study design, study location, number of years of follow-up, the mean age of participants, sex ratio (male/female) of participants, and qualitative evaluation score of articles were assessed.

In general, the odds ratio of stroke or hospitalization of the elderly in compared to nonvaccinated individuals, in the vaccinated group in cohort studies, was equal to 0.84 (95% CI: 0.77-0.90), in case-control studies was equal to 0.81(95% CI: 0.93-0.70), in North America was equal to 0.89(95% CI: 0.60-1.32), in Europe was equal to 0.79 (95% CI: 0.69 - 0.91), in Asia was equal to 0.83 (95% CI: 0.74-0.95), in people 70 years and older was equal to 0.82 (95% CI: 0.75-0.89), in people under 70 years was equal to 0.85 (95% CI: 0.73-0.99), in studies with more than or equal to 10,000 participants was equal to 0.84 (95% CI: 0.79-0.90), in studies with a number of participants less than 10,000 was equal to 0.70(95% CI: 0.49-1.01), in studies with a follow-up period of less than 60 months was equal to 0.84 (95% CI: 0.77-0.91), and in studies with follow-up period the same or more than 60 months was equal to 0.82 (CI: 95%: 0.67-1), in studies that were classified as good in terms of quality was equal to 0.88 (95% CI: 0.81-0.95), and in medium quality studies was equal to 0.70 (95% CI: 0.58-0.85), in studies with sex ratio (male to female) less than one was equal to 0.83(95% CI: 0.75-0.91), and in studies with sex ratio (male to female) the same or more than one was equal to 0.84 (CI: 95%: 0.72-0.97) (Table 4).

### 3.5. Evaluation of Publication Bias

In the study of the relationship between receiving the flu vaccine with stroke and its hospitalization in the elderly, using Begg's test (*P* value = 0.112) and Egger's test (*P* value = 0.490), no publication bias was observed. The corresponding funnel diagram can be seen in Figure 5.

## 4. Discussion

The purpose of this systematic review and meta-analysis study was to investigate the relationship between receiving the flu vaccine and the risk of stroke and hospitalization in the elderly. This study showed that compared to the nonvaccinated group, the OR of stroke or hospitalization in the vaccinated group is equal to 0.84 (95% CI: 0.77-0.90). In other words, the results of this meta-analysis show that compared with the elderly who did not receive the flu vaccine, the odds ratio of having a stroke or hospitalization was 16% lower for those who received the flu vaccine. Also, compared to the nonvaccinated people, the OR of having a stroke or hospitalization in the elderly in the age group less than 70 years is equal to 0.85 (0.73-0.99) and in the elderly 70 years and older is equal to 0.82 (0.75-0.89).

According to studies, infectious agents can increase the occurrence of stroke [47]. The systemic inflammatory response induced by influenza causes the rupture of vulnerable plaque through the concentration of reactive proteins and cytokines. The mechanism of these events is caused by impaired vasodilation by metabolic disorders and increased thrombotic tendencies by altered clotting factors and platelet dysfunction [48–50]. The immune response to vaccination may be another mechanism by which vaccination reduces the risk of stroke. Vaccine-induced antibodies activate the bradykinin-2 receptor and produce nitric oxide and dilate blood vessels, which may eventually lead to stabilization, atherosclerotic plaque, and reduced risk of CVD [51].

Atherosclerosis, plaque rupture, and vascular thrombosis can consider causes of stroke [20]. The role of infectious agents in atherosclerosis is well known. William Osler was one of the first to describe the role of infectious agents in the pathogenesis of atherosclerosis [52]. In the late 1970s, scientists began to study the role of herpes, chlamydia, or pneumonia and later Helicobacter pylori, Mycoplasma pneumonia, and Enterovirus into animal models and observed that these factors were associated with atherosclerosis [49, 50, 53–60]. These efforts coincided with the emergence of new evidence of atherosclerosis as an inflammatory disease [61]. Acute vascular syndrome involves the rupture of vulnerable plaques, which are usually nonconstructive and have a thin fibrous cap and a large fatty nucleus [62]. When the surface of these plaques ruptures or erodes, steroid thrombosis occurs. The factors that lead to plaque and inflammation are not fully identified. Accordingly, studies have hypothesized whether the flu may in some patients cause acute inflammation of the vascular wall and, with plaque instability, lead to acute vascular syndrome [60]. So, in influenza pandemics, deaths from CVD, hypertension, and stroke increased significantly [63–65].

A study conducted in 2014 by Lin et al. [43] showed that receiving the flu vaccine can reduce the risk of hospitalization. Influenza vaccination is one of the most effective ways to prevent stroke deaths, according to a 2017 meta-analysis by Lee et al. [35] on the effect of influenza vaccine on stroke risk; it was observed that the relative risk of stroke compared to unvaccinated individuals in vaccinated individuals is 0.75 (95% CI 0.82-0.91), which indicates that receiving the flu vaccine leads to a 25% reduction in the risk of occurrence of stroke. Studies by Lin Yang et al. [66] in 2019 and Puig-Barbera et al. [39] in 2007 also confirmed the protective effect of the flu vaccine against hospitalization of the elderly.

However, the results of some studies in this area are not in line with the results of the present study; for example, a study conducted by Ohmit and Monto [37] in 1995 in the US showed that the flu vaccine does not have a protective effect against hospitalization due to stroke, so the OR of hospitalization of vaccinated elderly is equal to 1.17 (95% CI: 0.73-1.88). Also, in another study conducted by Chang et al. [46] in 2020 in Taiwan, it was found that compared to the nonvaccinated group, the OR of hospitalization due to stroke in vaccinated elderly is equal to1.29 (95% CI: 1.22-1.36). Similarly, a study by Pinol-Ripoll et al. [40] in 2008 observed that the influenza vaccine in the elderly has no protective or risk factor effect against stroke, so OR of stroke in the nonvaccinated group was equal to 1.02 (95% CI: 0.77-1.36).

## 5. Limitations of the Study

This systematic review and meta-analysis study was conducted based on the results of research with case-control or cohort design, so it is necessary that in future studies the relationship between influenza vaccine and the occurrence of stroke and its hospitalization assessed based on the results of randomized clinical trial studies with appropriate sample size and adopting strict measures with long-term follow-up of people participating in the study.

In addition, in this study, it was not possible to analyze subgroups based on the type of vaccine received, because, in the studies included in the study, the type of vaccine received (injection/inhalation) in each study was not properly reported.

Moreover, the highest number of studies has been conducted in Asia, Europe, and North America, and no studies have been reported from Africa, South America, and Australia, so this problem can adversely affect the generalizability of the study results.

## 6. Conclusion

This systematic review and meta-analysis shows that receiving the flu vaccine can reduce the risk of stroke and its hospitalization in the elderly by 16% (10%-22%). Therefore, receiving this vaccine as a preventive intervention for stroke in the elderly may be promising.

## Figures and Tables

**Figure 1:** Diagram of selected studies for meta-analysis.

**Figure 2:** Forest plot of the relationship between receiving the flu vaccine with stroke and its hospitalization in the elderly.

**Figure 3:** Sensitivity analysis for the assessment of the relationship between receiving the flu vaccine with stroke and its hospitalization in the elderly.

**Figure 4:** Galbraith plot showing heterogeneity in meta-analysis studies.

**Figure 5:** Funnel plot for evaluation of publication bias in investigating the relationship between receiving the flu vaccine with stroke and its hospitalization in the elderly.

**Table 1:** Characteristics of meta-analysis studies to investigate the relationship between receiving the flu vaccine and the risk of stroke and its hospitalization in the elderly.

Publication first author	Year	Study setting	Study design	Sample size	OR	95 % CI	Follow-up time (month)	Quality assessment
Lin [43]	2014	Taiwan	Case-control study	3120	0.8	(0.64–0.98)	36	6.5
Nichol [30]	2003	USA	Cohort	146328	0.77	(0.66–0.89)	24	8
Vamos [45]	2016	England	Cohort	124503	0.82	(0.67–1)	84	5.5
Hung [41]	2010	Hong Kong	Cohort	36636	0.67	(0.54–0.83)	12	6
Chang [46]	2020	Taiwan	Cohort	2741403	0.88	(0.83–0.94)	24	9
Ohmit [37]	1995	USA	Case-control study	4487	1.17	(0.73–1.88)	24	7.5
Pinol-Ripoll [40]	2008	Spain	Case-control	786	1.02	(0.77–1.36)	12	7
Grau [31]	2005	German	Case-control	740	0.46	(0.28–0.77)	24	6.5
Lavallee P [29]	2002	France	Case-control	689	0.37	(0.15–0.87)	60	6.5
Smeeth [24]	2004	UK	Nested case-control	23188	0.86	(0.76–0.97)	48	7
Lavallee PC [42]	2014	International	Prospective cohort	22837	1.01	(0.88–1.17)	48	8
Wang [38]	2004	Taiwan	Cohort	21347	0.96	(0.79–1.17)	6	7.5
Puig-Barbera J [39]	2007	Spain	Case-control study	380	0.07	(0.01–0.48)	12	8
Siriwardena [44]	2014	UK	Case-control study	72202	0.8	(0.76–0.84)	12	7.5

**Table 2:** Adjusted variables in the studies that investigate the relationship between receiving the flu vaccine with stroke and its hospitalization in the elderly.

Publication first author	Year	Adjusted variables
Lin [43]	2014	Diabetes, hypertension, hyperlipidemia, coronary heart disease, atrial fibrillation, and chronic rheumatic Int. J. Environ. Res-heart disease
Nichol [30]	2003	Age, sex, and site
Vamos [45]	2016	Age, sex, index of multiple deprivation quintile, number of comorbid conditions, duration of diabetes, body mass index, smoking status, systolic and diastolic blood pressure, serum cholesterol and glycated hemoglobin, use of lipid-lowering drugs, anticoagulants or antiplatelet drugs, antihypertensive drugs, insulin, oral antihyperglycemic drugs or immunosuppressive drugs, number of hospital admissions during the previous year, history of pneumococcal vaccination, and influenza vaccination during the previous year and cohort year
Hung [41]	2010	—
Chang [46]	2020	Age, gender, premium salary, urbanization level, CCI score, catastrophic illnesses, status as long-term care facility resident, outpatient utilization, hospital admission, and utilization of health examination services
Ohmit [37]	1995	—
Puig-Barbera J [39]	2007	Lifestyle factors use of healthcare functionality propensity score nonseason data
Pinol-Ripoll [40]	2008	Lifestyle factors
Grau [31]	2005	Hypertension, alcohol abstinence, high alcohol consumption, and sports
Lavallee P [29]	2002	Age, sex, diabetes, hypertension, body mass index, current smoking, and cholesterol
Smeeth [24]	2004	Age
Lavallee PC [42]	2014	Propensity score
Wang [38]	2004	Pulmonary disease
Siriwardena [44]	2014	Chronic heart disease, asthma/COPD, diabetes, chronic renal failure, chronic liver disease, splenectomy, immunosuppression/HIV, Charlson (comorbidity) index, hypertension, peripheral vascular disease, hyperlipidemia, smoking status, family history of stroke/TIA, family history of AMI, aspirin uptake, antihypertensive treatment, statin uptake, number of home visits, and general practice consultation

**Table 3:** Results of sensitivity analysis for the assessment of the relationship between receiving the flu vaccine with stroke and its hospitalization in the elderly.

Lead author	Year	OR (95% CI)
Ohmit SE	1995	0.83 (0.76-0.89)
Wang CS	2004	0.83 (0.76-0.89)
Vamos EP	2016	0.84 (0.77-0.90)
Grau AJ	2005	0.85 (0.78-0.91)
Lin HC	2014	0.84 (0.77-0.92)
Hung IFN	2010	0.85 (0.79-0.92)
Nichol KL	2003	0.84 (0.78-0.92)
Lavallee PC	2002	0.84 (0.78-0.91)
Lavallee PC	2014	0.82 (0.76-0.89)
Pinol-Ripoll G	2008	0.83 (0.76-0.89)
Puig-Barbera J	2007	0.84 (0.78-0.90)
Siriwardena AN	2014	0.84 (0.76-0.92)
Smeeth L	2004	0.83 (0.76-0.91)
Chang YC	2020	0.83 (0.75-0.91)

**Table 4:** Subgroup analysis of the association between receiving the flu vaccine with stroke and its hospitalization in the elderly.

Characteristics		Number of studies	OR (95% CI)	*P* value	Heterogeneity
Study design	Cohort	6	0.85 (0.77-0.94)	0.017	63.8%
	Case-control	8	0.81 (0.70-0.93)	0.005	65.1%

Study location	North America	2	0.89 (0.60-1.32)	0.098	63.4%
	Europe	7	0.79 (0.69-0.91)	0.007	66.2%
	International	1	1.01 (0.88–1.17)	—	0.0
	Asia	4	0.83 (0.74-0.95)	0.061	59.2%

Average age	<70	9	0.85 (0.73-0.99)	≤0.001	73.2%
	≥70	5	0.82 (0.75-0.89)	0.095	49.4%

Follow up - time	Less than 5	13	0.84 (0.77-0.91)	≤0.001	68.6%
	More than 5	1	0.82 (0.67-1.00)	—	0.0%

Sample size	Less than 10,000	6	0.70 (0.49-1.01)	0.002	73.5%
	More than 10,000	8	0.84 (0.79-0.90)	0.007	63.7%

Quality assessment	Good quality	9	0.88 (0.81-0.95)	0.002	68.1%
	Medium quality	5	0.70 (0.58-0.85)	0.084	51.3%

Sex ratio (male to female)	Less than one	7	0.83 (0.75-0.91)	≤0.001	70.9%
	Equal or more than one	7	0.84 (0.72-0.97)	0.021	63.4%

## Data Availability

The data used in this systematic review and meta-analysis can be retrieved in the tables provided in the text of the article. In addition, the data used for meta-analysis in the present study is freely available in the text of the articles used.
